# Leg Stiffness and Vertical Stiffness of Habitual Forefoot and Rearfoot Strikers during Running

**DOI:** 10.1155/2020/8866340

**Published:** 2020-11-24

**Authors:** Lulu Yin, Xiaoyue Hu, Zhangqi Lai, Kun Liu, Lin Wang

**Affiliations:** ^1^Department of Critical Care Medicine, Shanghai Tenth People's Hospital, School of Medicine, Tongji University, Shanghai, China; ^2^School of Kinesiology, Shanghai University of Sport, Shanghai, China; ^3^Department of Rehabilitation Medicine, Shanghai Jiao Tong University Affiliated Sixth People's Hospital, Shanghai, China

## Abstract

Foot strike patterns influence the running efficiency and may be an injury risk. However, differences in the leg stiffness between runners with habitual forefoot (hFFS) and habitual rearfoot (hRFS) strike patterns remain unclear. This study aimed at determining the differences in the stiffness, associated loading rate, and kinematic performance between runners with hFFS and hRFS during running. Kinematic and kinetic data were collected amongst 39 runners with hFFS and 39 runners with hRFS running at speed of 3.3 m/s, leg stiffness (Kleg), and vertical stiffness (Kvert), and impact loads were calculated. Results found that runners with hFFS had greater Kleg (*P* = 0.010, Cohen′s *d* = 0.60), greater peak vertical ground reaction force (vGRF) (*P* = 0.040, Cohen′s *d* = 0.47), shorter contact time(*t*_*c*_) (*P* < 0.001, Cohen′s *d* = 0.85), and smaller maximum leg compression (Δ*L ***)** (*P* = 0.002, Cohen′s *d* = 0.72) compared with their hRFS counterparts. Runners with hFFS had lower impact peak (IP) (*P* < 0.001, Cohen′s *d* = 1.65), vertical average loading rate (VALR) (*P* < 0.001, Cohen′s *d* = 1.20), and vertical instantaneous loading rate (VILR) (*P* < 0.001, Cohen′s *d* = 1.14) compared with runners with hRFS. Runners with hFFS landed with a plantar flexed ankle, whereas runners with hRFS landed with a dorsiflexed ankle (*P* < 0.001, Cohen′s *d* = 3.35). Runners with hFFS also exhibited more flexed hip (*P* = 0.020, Cohen′s *d* = 0.61) and knee (*P* < 0.001, Cohen′s *d* = 1.15) than runners with hRFS at initial contact. These results might indicate that runners with hFFS were associated with better running economy through the transmission of elastic energy.

## 1. Introduction

Running, a prevalent and convenient aerobic exercise, improves physical fitness and psychological health [1]. However, the incidence of running-related injuries (RRIs) in the lower extremities ranges from 19.4% to 79.3% during long-distance running because of the repeated loading of the musculoskeletal system [2]. RRI-related risk factors include previous injuries, weekly distance and frequency [3], running surface [4], footwear condition [5], and foot strike pattern [6].

The foot strike pattern is an important factor that affects the running performance and the occurrence of sports injury. The foot strike pattern is categorised generally into rearfoot (RFS), midfoot (MFS), and forefoot (FFS) strikes, which depend on the center of pressure relative to a foot that initially contacts the running ground [7]. The RFS is the most prevalent foot strike pattern with more than 75% elite runners [8], and 85% recreational runners [9] are reported to adopt the RFS pattern. However, FFS exhibited lower impact collisions at initial contact according to previous research [10]. At present, numerous running coaches have trained runners with hRFS transforming into hFFS. Therefore, the underlying mechanism of different foot strike patterns should be clarified to provide evidence-based recommendation for runners.

Numerous studies have explored the biomechanical differences from spatial–temporal features, kinematic variables, kinetic variables, and muscle activity between RFS and FFS. The RFS lands with the dorsiflexed ankle, thereby exposing an impact peak of about 1.6 body weight (BW) during early stance and transmitting more axial vGRF to the knee [11]. Therefore, the RFS is demonstrated to be associated with patellofemoral disorders [12]. By contrast, the FFS lands with the plantar flexed ankle without the visible IP of GRF [10] accompanying the greater eccentric contraction in the triceps surae [13]. Consequently, this pattern exhibits a compliant ankle to absorb the impact force and reduces the associated loading rate [6, 11]. However, the excessive contraction in ankle plantar flexion muscles can increase the risk of the Achilles tendinopathy in FFS ([14]; H. [15]).

The spring–mass model is frequently used to describe the spring-like compression of the leg loaded by the body mass and reflects the general mechanisms on how the whole lower limb, including joints, muscles, tendons, ligaments, and bones, coordinate to cope with an external impact, transmit elastic potential energy, and subsequently rebound [16]. Few studies have explored running features in terms of the foot strike pattern from a holistic view. During running, leg stiffness is defined as the ratio of the peak vGRF to the maximum leg compression, and vertical stiffness is defined as the ratio of the peak vGRF to the vertical center of mass (COM) displacement (Δ*y*_*c*_) [17]. These variables are calculated from the time–vGRF curve and used mostly to reflect the storage and the reutilization of the elastic energy of the lower leg. Previous studies confirm that a stiff leg may facilitate the efficient storage and reutilization of elastic energy, thereby enhancing the athletic performance in stretch–shortening cycles during running [18]. The Kleg and the Kvert play an important role during running efficiency, but limited evidence is available regarding the effect of the foot strike pattern on stiffness during running [19, 20].

Therefore, this study aimed at determining the difference on the Kleg and the Kvert and corresponding components, including peak vGRF, *t*_*c*_, Δ*L*, and Δ*y*_*c*_ between runners with hRFS and hFFS during running. For comprehensive interpretation, the associated IP, loading rate, and the joint sagittal angle of the lower extremity at initial contact are also investigated. This study hypothesises the following: (1) the Kleg and the Kvert of runners with hFFS are higher than those of runners with hRFS. (2) Compared with runners with hRFS, runners with hFFS have a more flexed sagittal angle of the lower limb joint at initial contact and lower IP and loading rate.

## 2. Materials and Methods

### 2.1. Participants

Considering an effect size (ES) of 0.70, power of 0.80, and *α* level of 0.05, a minimum of 34 participants wasrequired for each group. Finally, 39 participants in each group were recruited in this research to avoid missing data. Male healthy amateur runners with hRFS (*n* = 39, age = 24.1 ± 2.4 years, height = 172.4 ± 5.8 cm, weight = 69.0 ± 10.4 kg, running experience = 2.9 ± 2.0 years) and hFFS (*n* = 39, age = 28.3 ± 6.8 years, height = 173.1 ± 4.3 cm, weight = 67.6 ± 9.6 kg, running experience = 4.3 ± 3.6 years) were recruited from a local university and running clubs. The participants ran regularly for 10–15 km per week for at least six months. Foot strike patterns were determined using the Novel Pedar-X system (Novel, Munich, Germany) in advance sampling at 100 Hz to identify the position of the pressure center during running in the customary landing style and the self-selected velocity of participants. On the initial foot landing, the participants whose foot center of pressure was located in the anterior third of the foot were included in the hFFS group, and the participants whose foot center of pressure was located in the posterior third of the foot were placed in the hRFS group [7]. Runners who landed with a midfoot strike landing pattern were excluded because the MFS pattern was highly different from the FFS and the RFS patterns [10]. Flat feet, high arched feet, and other foot deformations were also excluded. All participants had to be right-leg dominant, which was verified by kicking a ball. The participants did not have a history of musculoskeletal problems, such as a recent injury or surgery in the past six months or any disease that could affect their running condition, and signed an informed consent form. This study was approved by the Ethics Committee of the Shanghai University of Sport.

### 2.2. Experimental Protocol

Experiments were conducted in our laboratory through 3D motion analysis with ten cameras (Vicon T40, Oxford Metrics, UK). A total of 23 reflective markers were placed on the participants' bony landmarks based on the full-body Plug-in Gait Model at an acquisition sampling rate of 200 Hz. Two 3D force platforms (Kistler Instruments Corp. Switzerland) synchronised with the motion capture system were used to collect the ground reaction force data at 2000 Hz.

A rubber runway with a length of 15 m, a width of 1 m, and a thickness of 2 cm was constructed in our laboratory to simulate an outdoor rubber track. All participants wore uniform socks and lightweight running shoes (Asics TM467) without thick heels and additional cushioning structures to ensure no interference with running characteristics [21].

The participants warmed up on a treadmill for 15 min by using their habitual foot strike pattern at their self-selected speed and performed practice trials on the rubber runway to be familiar with the experimental environments. During practice, the participants were instructed to maintain a consistent running velocity at 3.3 m/s (±5%) confirmed by an optical fibre door and to make contact with the central portion of the force platform with their right foot without deliberately modifying their gait. Three successful trials were then collected for each subject.

### 2.3. Data Analysis

Data were processed in the Visual 3D (C-Motion, Rockville, MD, USA). A pelvis and three-segment lower limb plug-in gait model (i.e., thigh, shank, and foot) was constructed to determine the sagittal joint angles of the hip, knee and ankle joints, and COM trajectory of the hFFS and the hRFS groups. Data were filtered using a fourth-order low-pass Butterworth filter with a cut-off frequency (kinematics:10 Hz; GRFs:50 Hz) [22]. The initial contact was defined as the moment when the vGRF data first became greater than 20 N, and toe off was defined after the vGRF data became lower than 20 N.

Kleg (kN/m) was calculated as the ratio of the peak vGRF to the Δ*L* during the stance phase as follows [19]:

(1) $$\begin{array}{c} \text{Kleg}=\frac{{vGRF}_{\text{peak}}}{\Delta L},\text{wit}h\;\Delta L=\Delta y_{c}+L_{0}-\sqrt{L_{0}^{2}-{\left(\frac{1}{2}vt_{c}\right)}^{2}}, \end{array}$$

where the Δ*L* is the maximum vertical variation of the leg length during running, *L*_0_ is the leg length measured as the distance from the trochanter major to the prominence of the lateral malleolus when subjects stand upright with two feet, and *t*_*c*_ is the contact time during the stance phase when the vGRF is above the 20 N threshold.

Kvert (kN/m) was calculated as the ratio of the peak vGRF to the maximum Δ*y*_*c*_ during the stance phase as follows [19]:

(2) $$\begin{array}{c} \text{Kvert}=\frac{{vGRF}_{\text{peak}}}{\Delta y_{c}}. \end{array}$$

VALR, VILR, and IP were determined from the time–vGRF curve. The VALR was calculated as the total change in the vGRF divided by the total change in time within 20%–80% between the foot strike and the IP. The VILR was the peak sample-to-sample loading rate occurring during the same period [23, 24]. In case FFS whose IP was absent from the vertical GRF curve, the force value at 13% of the stance was used [24]. All GRF variables were normalised to the BW.

### 2.4. Statistical Analysis

Data were presented as mean and standard deviation. The Shapiro–Wilk and the Levene tests were performed to confirm the normal distribution and the equality of variances, respectively. An independent *t*-test was conducted to compare leg and vertical stiffness, impact variables, and sagittal angles of hip, knee, and ankle at initial contact. The ES was calculated using Cohen's *d*. Values of 0.2 ≤ *d* < 0.5, 0.5 ≤ *d* < 0.8, and *d* > 0.8 represented small, medium, and large differences, respectively. The statistical significance was set at *P* < 0.05. Statistical analysis was performed using the SPSS version 20.0 (IBM, Chicago, IL, USA).

## 3. Results

As shown in Table 1, the Kleg of runners with hFFS was 12.7% higher (*P* = 0.010, Cohen′s *d* = 0.60) than that of runners with hRFS. Compared with runners with hRFS, runners with hFFS had 8% lower contact time (*P* < 0.001, Cohen′s *d* = 0.85), 10% less Δ*L* (*P* = 0.002, Cohen′s *d* = 0.72), and 4.2% higher vGRF_peak_ (*P* = 0.04, Cohen′s *d* = 0.47). However, the Kvert and the Δ*y*_*c*_ of runners with hRFS did not significantly differ from those of runners with hFFS.

For impact variables, the IP (*P* < 0.001, Cohen′s *d* = 1.65), VALR (*P* < 0.001, Cohen′s *d* = 1.20), and VILR (*P* < 0.001, Cohen′s *d* = 1.14) of runners with hFFS were 42.64%, 79.74%, and 64.42% lower, respectively, than those of runners with hRFS.

For sagittal angles at initial contact, the hip (*P* = 0.020, Cohen′s *d* = 0.61) and the knee (*P* < 0.001, Cohen′s *d* = 1.15) of runners with hFFS were 15.9% and 40.3% more flexed, respectively, than those of runners with hRFS. Runners with hFFS landed with a plantar flexed ankle (−14.58° ± 6.38°), whereas runners with hRFS landed with a dorsiflexed ankle (8.53° ± 4.60°). These findings significantly differed (*P* < 0.001, Cohen′s *d* = 4.15).

## 4. Discussion

This study has investigated Kleg, Kvert, associated loading rates, and joint angle differences at initial contact between runners with hRFS and hFFS. Stiffness represents the resistance of body to coping with the applied force to prevent lower limb collapse, thereby modulating running-related [25] and injuries [19].

Partly consistent with hypothesis, results have indicated that runners with hFFS have greater Δ*L* and peak vGRF and shorter contact time, thereby resulting in greater Kleg, than runners with hRFS. However, runners with hRFS and hFFS show no significant difference in the Δ*y*_*c*_ and the Kvert. According to previous research [20], the Kleg is used generally to describe horizontal and vertical movement features, such as running and directional jump, whereas the Kvert is used generally to describe the linear motion efficiency with simple vertical direction, such as the vertical jump of double feet and single foot. Therefore, the Kleg is possibly more sensitive than the Kvert [26] in representing the running efficiency in this study because of the horizontal–forward movement property of running, and the vertical and frontal displacements of COM approach the sine curve [20].

Our results indicate that the Kleg of runners with hFFS is 12.7% greater than that of runners with hRFS. This result demonstrated that hFFS might be advantageous for the running efficiency through a relatively stiff rebound and high force production and transmission during the stance phase [20, 27, 28]. The stiffness refers to the joint excursion in response to impulse loading applied to the bone and the cartilage. Although studies have speculated that stiffness and injuries might be related [18, 29], the interrelationship between the Kleg and the injury risk remains unclear.

The contact time is considered the most sensitive parameter and has approximately a 1 : 2 negative effect on Kleg; that is, a 10% decrease in contact time leads to about 20% increase in Kleg [17, 30]. In this study, compared with runners with hRFS, runners with hFFS may produce higher level precontraction before contact, and the accumulated sufficient tension in lower limbs regulates the Kleg during the short-distance running.

Moreover, our results indicate that the Kvert and the Δ*y*_*c*_ of runners with hRFS and hFFS do not significantly differ. This finding is consistent with the observations of Shih [5], who has found no significant difference in the Kvert between the RFS and the FFS in barefoot and shod running. Changes in Kvert are possibly attributed to alterations in the displacement of COM [31]. This study suggests that runners with hRFS and hFFS can adjust their strategies to optimise the oscillation of COM to minimize the energy consumption (D. S. [32]).

Unsurprisingly, consistent with previous research, the impact variables [24, 33–36], IP, VALR, and VILR of runners with hFFS, are lower than those of runners with hRFS. The IP and the loading rate are intuitional to reflect the impact transmitting to the body and associated sensitively with the injury rate [37]. During the early-stance phase, runners with hFFS land with the plantar flexion ankle and turn to the dorsiflexion [36]. During this process, participants experienced a multisegment cushion from the forefoot to the calcaneus, and the mechanical work is performed using the intrinsic foot muscles [38]. The plantar flexed ankle absorbs increased energy through the eccentric control of triceps surae [39]. However, too much ankle plantar flexor moment can lead to Achilles tendinopathy [13], and too much load in the forefoot region can lead to metatarsal stress fractures [40]. By contrast, runners with RFS land with their heel without the cushion effect, like FFS, transmitting increased axial force along the shank to the knee and contributing to increased IP and loading rate. However, the energy absorption, which demands increased eccentric control by quadriceps in runners with hRFS, concentrates in the knee joint. However, the excessive contraction of quadriceps may be associated with the patellofemoral pain syndrome [24].

In terms of the kinematic parameters at the initial touch down, results indicate that runners with hFFS have a plantar flexed ankle and more flexed hip and knee compared with runners with hRFS. These findings are consistent with those of previous studies [5, 13, 41]. During the early stance, runners with hFFS maintain the ankle position in the plantar flexion through an earlier and longer eccentric contraction in the triceps surae than runners with hRFS [5, 13, 36]. This process can provide a cushion effect to alleviate the transient impact, thereby reducing the knee joint contact force and risks of knee injuries, such as patellofemoral pain and tibial stress fracture [6, 11, 23].

The hip and the knee are flexed to minimize the displacement of COM and offset the potential increased Δ*y*_*c*_ in hFFS. On the horizontal plane, the more flexed hip and knee may increase the trunk forward lean and decrease the distance from the landing position to the projection of COM (D. S. Williams, 3rd et al., 2012) and consequently provide improved cushion effect. However, a large distance from the landing position to the projection of COM in FFS is observed by Williams (D. S. [32]) and Shih [5], and this finding is likely because participants in their studies have run with the acute transition to FFS. The muscle architecture and the neuromuscular control have not adapted to the FFS pattern [42].

Notably, the participants in this study have used their habitual foot strike pattern, which is different from the immediate transition from RFS to FFS in previous studies [5, 33, 36]. According to motor learning [42], the process of transition for the foot strike pattern gets through the “transition period” when the muscular structure and the motor strategy adapt gradually to the new foot strike pattern. Therefore, the runners with their preferred running mode in our study avoid the cofounding effect of the “transition period”, providing intuitive view to compare the biomechanic differences between runners with hFFS and hRFS.

### 4.1. Limitations

Limitations need to be considered when interpreting the results. Firstly, the Kleg and the Kvert are calculated from vGRF and Δ*y*_*c*_, and the sagittal nature makes it insufficient to completely represent the mechanics of running, which is a three-dimensional locomotion. As such, results should be cautiously interpreted. Secondly, Kleg and Kvert measurement is executed in the stance phase during short-distance running. However, describing the dynamic stiffness fluctuation with different running distances, surfaces, and slopes in an actual environment is difficult.

## 5. Conclusions

This study indicated that compared with runners with hRFS, runners with hFFS have a higher Kleg, corresponding shorter contact time and lower Δ*L* during the stance phase. Moreover, runners with hFFS land with a more flexed lower limb and have a lower IP and loading rate. These results may indicate that runners with hFFS are associated with better running economy through the transmission of elastic energy.

## Figures and Tables

**Table 1:** Comparison of leg and vertical stiffness, impact parameters, and sagittal angles at initial contact between runners with hRFS and hFFS (mean ± standard deviation).

	hRFS	hFFS	*P* values	Cohen's *d*
Stiffness parameters				
Kleg(KN/m)	8.84 ± 1.78	9.96 ± 1.97	0.010^∗^	0.60
Kvert(KN/m)	20.65 ± 3.97	21.32 ± 3.35	0.418	0.18
*t*_*c*_ (s)	0.25 ± 0.02	0.23 ± 0.02	<0.001^∗^	0.85
Δ*L* (m)	0.20 ± 0.03	0.18 ± 0.03	0.002^∗^	0.72
Δ*y*_*c*_ (m)	0.09 ± 0.01	0.09 ± 0.01	0.511	0.15
vGRF_peak_(BW)	2.61 ± 0.20	2.72 ± 0.23	0.040^∗^	0.47
Impact parameters				
IP (BW)	1.84 ± 0.36	1.29 ± 0.30	<0.001^∗^	1.65
VALR (BW/s)	160.67 ± 73.11	89.39 ± 40.92	<0.001^∗^	1.20
VILR (BW/s)	226.84 ± 95.77	137.96 ± 55.25	<0.001^∗^	1.14
Sagittal angles at initial contact				
Hip	41.76 ± 11.08	48.40 ± 10.86	0.020^∗^	0.61
Knee	14.02 ± 4.39	19.67 ± 5.40	<0.001^∗^	1.15
Ankle	8.53 ± 4.60	−14.58 ± 6.38	<0.001^∗^	4.15

MD: mean difference; CI: confidence interval; Kleg: leg stiffness; Kvert: vertical stiffness; *t*_*c*_: contact time; Δ*L*: maximum leg compression during stance; Δ*y*_*c*_: vertical displacement of the center of mass during stance; vGRF peak: peak vertical ground reaction force; IP: impact peak; VALR: vertical average loading rate; VILR: vertical instantaneous loading rate. ^∗^ means with significant difference between runners with hRFS and hFFS (*P* < 0.05).

## Data Availability

We have uploaded our raw data and approval of Ethics Committee in Dryad, Dataset, 10.5061/dryad.d2547d7z4. You can visit dataset files with others using the URL (https://datadryad.org/stash/share/ZDAvL8jlao-YkcWrsaFl7g1qjFqNyvrM1xCrdLxesCE).
